RETRACTED

# Flavor and Rapid Prediction of Red Wine by the Chemometrics Algorithm Based on Multidimensional Spectral Data

**DOI:** 10.1155/2022/1418022

**Published:** 2022-08-04

**Authors:** Qiao Wu

**Affiliations:** Department of Pharmacy, Changsha Health Vocational College, Changsha 410100, Hunan, China

## Abstract

Since its birth, red wine has been loved by people of all walks of life. The taste of red wine has changed and the pursuit of quality has always been the most sought-after goal by sommeliers, winemakers, and the public. However, due to the rich taste of red wine, any link is willing to produce different flavors. At present, there is no quantitative control study on the flavor of red wine. The purpose of this paper is to analyze the flavor of red wine through the chemometric algorithm and establish a reasonable model to predict the flavor of red wine. Aiming at the research of red wine flavor, this paper designs a red wine flavor extraction experiment and extracts the substances that produce an aroma and flavor in red wine to the greatest extent through strict selection of extraction head and reaction time. For the rapid analysis of red wine flavor, this paper quantitatively describes the chemical category, volatilization time, molecular weight, etc., of flavor substances by analyzing the multidimensional spectral data of red wine, so that flavor substances can be quickly located. The experimental results of this paper prove that, for different red wines, the algorithm in this paper can accurately identify the flavor substances in red wine. Also, for red wine multidimensional spectral data, the algorithm in this paper can improve the accuracy by 30% and save the running time by 30%. This shows that the research in this paper can analyze and quickly predict the flavor of red wine.

## 1. Introduction

The taste of the wine, as well as the color and aroma of the wine, are important indicators for evaluating the quality of a wine. After wine enters the mouth, it will produce sensory reactions such as acid, thorn, astringency, bitterness, balance, suppleness, and viscosity. These evaluations come from the sensory nerve cells on the human taste buds. The texture of the wine body mainly comes from the ethanol, glycerol, residual sugar, polysaccharide, carbon dioxide, and polyphenols in the wine, which are the comprehensive evaluation indicators produced by the interaction with the taste buds in the mouth. Most of the current research focuses on the research on the aroma components of wine, and the research on the taste of wine, and the physiological response of people's oral cavity is relatively lacking. Therefore, the chemometrics algorithm based on multidimensional spectral data analysis is necessary for red wine flavor analysis and rapid prediction research.

RETRACTED

The content of wine aroma components in wine is less than 1%, but it determines the quality and quality of wine. There are many studies on the aroma components of distilled spirits, and the aroma components of distilled spirits with different types of raw materials are different. There are many studies on the wine aroma. Among them, Kong et al. designed a mixed fermentation process of Pichia and *Saccharomyces cerevisiae* for the problem of the weak aroma in thorn wine [1]. The focus of the Manuel research is to provide the latest knowledge and practices in preventing this problem in the wine industry [2]. The objective of Schumaker was to evaluate the effect of three wine flavor matrices on consumer acceptance and the temporal sensory properties of wines containing high and low concentrations of Brettanomyces metabolites [3]. Luca et al. aimed to examine how music affects wine flavor. His findings found that Chardonnay wines were perceived as more refined and sweeter when accompanied by a classical music background. On the other hand, in the case of Merlot, it is perceived as less alcohol when high volume pop music is delivered [4]. Khalilova et al. presented the results of research on fatty acids and antibacterial properties in red wine [5]. Carpenter et al. used Brussels sprouts as a typical bitter vegetable and studied some of the different effects [6]. The aroma of wine is the most important factor of wine flavor, but related scholars are mostly improving its production process, and there are relatively few studies on flavor chemicals, and there is no corresponding mathematical model to summarize.

Chemometric algorithms have important applications in chemical analysis, and there are many studies on them. Sun used four classifiers for hyperspectral imaging of peach chilling injury classification. He studied and compared three chilling damage classification schemes [7]. Lukasz resolved fluorescence spectra of three-component systems. He used rank annihilation factor analysis to determine the Stern-Volmer constant. It is a derivation of the modified Stern-Volmer formula in the case of differential fluorescence spectroscopy [8]. Jin et al. believed that electrothermal evaporation has been used for some time as an alternative sample introduction method in atomic spectroscopy, and due to its high sensitivity and efficient separation of analytes from matrix materials. It provides a better solution for the rapid analysis of complex samples [9]. Huang et al. explored the possibility of using hyperspectral imaging technology combined with chemometrics to rapidly and non-destructively predict anthocyanin content and antioxidant activity in mulberry [10]. It can be found that most of the related studies are the control variables of the experimental control group to analyze the source of the aroma and optimize them, but there is a lack of quantitative analysis of mathematical models. Therefore, this paper will quantitatively analyze and predict the flavor of red wine.

RETRACTED

For the flavor of red wine, the volatilization time of alcohols, acids, and lipids in the fermentation process is about 20 min, and the trend is the same, which shows that the prediction of red wine flavor can be predicted from the volatilization time of alcohols, lipids, and acids. The innovations of this paper are as follows: the improved frequency-domain extraction method of dynamic spectrum based on short-time Fourier transform (STFT) mainly starts from making up for the lack of time-varying information in fast Fourier transform (FFT). It combines the short-time Fourier transform with the Pauta criterion, which fully reflects the time-variation of the spectral signal in the frequency domain, and at the same time eliminates the corresponding replacement of the singular values in the signal. The utilization rate of the effective information of the spectral data is greatly improved, and the stability and accuracy of the model in the later prediction process of the hemoglobin concentration are enhanced.

## 2. Working Principle of Red Wine Flavor

### 2.1. Red Wine Flavor

In the brewing process of wine, alcoholic fermentation is accompanied by 1.5–2% sugars, which will ferment and produce by-products. There are many types of by-products. It includes esters, alcohols, acids, aldehydes, and sulfides, among others. The proper amount, content, and proportion of these by-products constitute the harmonious and harmonious flavor of the wine.

Alcohols are the metabolites of yeast in the fermentation process, and the main components are ethanol and other trace amounts of higher alcohols. Alcohol plays a great role in wine as a whole and has an important impact on the overall quality of wine. Higher alcohols are the main aroma substances in wine, and trace amounts of higher alcohols can enrich the taste and highlight the characteristic aroma of wine [11, 12].

Esters are the products of yeast fermentation and aromatic compounds produced during the aging process, which are the most important contributors to the ideal fermentation aroma. The fruity odors produced by fermentation are characterized by apple-flavored hexyl acetate and ethyl caprylate. It is a mixture of isoamyl acetate with banana flavor and phenethyl acetate with honey, fruit, and flower flavors. The presence of esters enriches the aroma of different fruit raw materials, improves the aroma and taste, and gives the wine a special aroma. During the fermentation process of red wine, in addition to yeast metabolism producing a variety of flavor substances, Monascus can produce abundant enzymes, volatile substances, pigments, and other metabolites. It gives red wine a different flavor than ordinary wine. The aroma transformation of the wine is shown in Figure 1. Flavor metabolites in wine fermentation are shown in Figure 2.

RETRACTED

The final flavor of a wine is the result of complex interactions between chemical components and specific fermentation conditions, such as temperature. The chemical composition of wine mainly depends on the variety and quality of fermented raw materials. Taking wine as an example, its aroma and flavor are closely related to the cultivation and the brewing process of grapes. The cultivation of grapes mainly focuses on individual cultivation of the flavor and the aroma of a high-quality grape variety in a special area. When brewing, it needs to be specially processed according to the picking time, maturity, and fermentation process. Except for a small part of prefermentation treatment, the microbial population of the remaining grapes, the selection of wine-making bacteria, and the process of malolactic fermentation have significant correlation with the aroma and flavor of wine. Even the final filtration and aging can affect the aroma and flavor of the wine [13].

### 2.2. Dynamic Spectrum Extraction Method Based on Short-Time Fourier Transform

The dynamic spectral frequency-domain extraction method is an extraction method based on fast Fourier transform. Its extraction results can only show every frequency contained in the noisy PPG signal. It cannot obtain the specific generation time and duration of the noise signal, so it cannot be eliminated or corrected. To solve this problem, a dynamic spectrum extraction method based on short-time Fourier transform is proposed in this paper.

In the process of converting the signal from the time domain to the frequency domain for analysis, since the traditional Fourier transform needs to use all the time domain information of the signal, it does not reflect the change of the frequency component of the signal with time. The singular value in the signal cannot be detected more accurately. In view of the above shortcomings, the rectangular window function *g*(*t*) shown in formula (1) is proposed. This paper uses the window function to segment the original logarithmic photoelectric pulse wave signal. At the same time, let the window slide with a certain step size *u*, and perform Fourier transform on the original signal segment in the window function after each sliding, according to the principle of 3 *σ* criteria [14, 15]. It detects and rejects (replaces) “singular values” in the sub-PPG signal. This dynamic spectral extraction method is called the short-time Fourier transform method.

RETRACTED

Rectangular window function formula is

(1) $$\begin{array}{c} g\left(t\right)=\left\{\begin{array}{cc} 1, & t_{s}\leq t\leq t_{e}\\ 0, & \text{else} \end{array}\right.. \end{array}$$

Among them, *t*_*s*_ represents the position of the data starting point of the window function in the original data time domain, *t*_*e*_ represents the position of the data end point of the window function in the original data time domain, and the difference between the two is the window function length.

The dynamic spectrum extraction formula based on short-time Fourier transform is

(2) $$\begin{array}{c} {\text{DS}}_{ij}=kX_{ij}\left(1\right),i=1,2,\ldots ,m;j=1,2,\ldots ,n. \end{array}$$

Among them, *m* represents the number of segments divided by the original spectral data after short-time Fourier transform, *n* represents the number of wavelengths, and DS_*ij*_ is the dynamic spectral value of the *i*th segment logarithmic photoplethysmography signal at the *j*th wavelength. *X*_*ij*_(1) represents the fundamental component of the *i*th pulse wave signal at the *j*th wavelength after short-time Fourier transform. *k* is the scaling factor between the dynamic spectral signal and the amplitude of the fundamental component of the original signal.

### 2.3. Dimensionality Reduction Based on Sparse Graph Learning

Figure 3 is a schematic flowchart of the learning process of SGL-DR based on dimensionality reduction based on sparse graph learning (SGL-DR). In this subsection, the proposed SGL-DR will be introduced in detail. SGL-DR is mainly divided into two parts, the first part is to use empty spectral clustering to divide all the data into K subsets. The second part is to obtain the final required projection matrix by iteratively learning the sparse graph and the projection matrix. Due to the use of clustering in the first part, the construction process of the sparse graph can be divided into the construction of K subgraphs, which can reduce the time cost of sparse representation without reducing the experimental effect.

In sparse graph construction, each pixel is represented by a small number of pixels by minimizing the sum of the reconstruction error and the sparse regularization term. Although the sparse graph has some advantages due to its sparse representation, it is also affected by the spectral similarity of different objects. In the work of this chapter, some additional useful information will be added to the sparse representation solution process, resulting in more efficient sparse graphs. Therefore, a new sparse graph learning framework is proposed with the corresponding objective function as the following formula:

(3) $$\begin{array}{c} \underset{P,\Theta }{\min}\sum_{i=1}^{n}\sum_{j=1}^{n}\left(\left(1-\beta \right)w_{ij}^{\text{spa}+\text{spa}}+\beta w_{ij}^{\text{pro}}\right)\theta_{ij}. \end{array}$$

Among them,

(4) $$\begin{array}{c} {\left\|X-X\Theta \right\|}_{F}^{2}\leq \varepsilon ,\\ w_{ij}^{pro}={\left\|P^{T}x_{i}-P^{T}x_{j}\right\|}_{2},\\ w_{ij}^{\text{spa}+\text{spa}}=\alpha {\left\|\text{index}\left(x_{i}\right)-\text{index}\left(x_{j}\right)\right\|}_{2}+\left(1-\alpha \right){\left\|x_{i}-x_{j}\right\|}_{2},\\ \theta_{ii}=0\text{ and }\theta_{ij}\geq 0,\\ 0\leq \alpha \leq 1;\text{ and };0\leq \beta \leq 1. \end{array}$$

Among them, *w*_*ij*_^*pro*^ is the projection weight, which is determined by the distance between *x*_*i*_ and *x*_*j*_ in the projection space, and *w*_*ij*_^spa+spa^ is the space spectral weight, which is obtained by the weighted summation of the spatial distance and the inter-spectral distance of the pixel pair. *α* and *β* are two tuning parameters that control the influence of various information in the sparse graph learning process.

RETRACTED

In formula (3), there are two unknown variables (Θ and P) to be optimized, and an alternate iterative approach is used to solve them. Given one variable, it solves for the other variable. The detailed process of the optimization solution is given below.

First step is

(5) $$\begin{array}{c} w_{ij}=\left(1-\beta \right)w_{ij}^{\text{spa}+\text{spa}}+\beta w_{ij}^{\text{pro}}. \end{array}$$

Bringing formula (5) into formula (3) and transforming it into an unconstrained lasso problem, we get

(6) $$\begin{array}{c} \underset{\Theta }{\min}{\left\|X-X\Theta \right\|}_{F}^{2}+\lambda \sum_{i=1}^{n}\sum_{j=1}^{n}w_{ij}\theta_{ij}. \end{array}$$

Among them, *λ* is a sparse regularization parameter, which can adjust the sparsity of the sparse representation coefficient. The larger the *λ*, the sparser the result. Since the weights are introduced in formula (5), we need to use the weighted lasso's solution algorithm to solve.

In the second step, given Θ, formula (3) can be simplified to the following form:

(7) $$\begin{array}{c} \underset{P}{\min}\sum_{i=1}^{n}\sum_{j=1}^{n}{\left\|P^{T}x_{i}-P^{T}x_{j}\right\|}_{2}\theta_{ij}. \end{array}$$

The projection matrix *P* can be obtained by solving the formula. The formula can be converted into a more concise expression by the following transformation.

(8) $$\begin{array}{c} Tr\left[P^{T}X\left(\sum_{i=1}^{n}\sum_{j=1}^{n}\left(e_{i}-e_{j}\right){\left(e_{i}-e_{j}\right)}^{T}\theta_{ij}\right)X^{T}P\right]. \end{array}$$

Among them, *e*_*i*_ is a column vector of length *m*, only the ith atom is 1, and the rest are 0.

(9) $$\begin{array}{c} \sum_{i=1}^{n}\sum_{j=1}^{n}\left(e_{i}-e_{j}\right){\left(e_{i}-e_{j}\right)}^{T}\theta_{ij}=D_{\text{row}}+D_{\text{column}}-\Theta -\Theta^{T}. \end{array}$$

*D*_row_ is a diagonal matrix with row summed values of Θ as diagonal elements.

(10) $$\begin{array}{c} D_{\text{row}}=\text{diag}\left(\sum_{j=1}^{n}\Theta_{:j}\right). \end{array}$$

*D*_column_ is the value of the column summation of Θ as a diagonal matrix of diagonal elements:

(11) $$\begin{array}{c} D_{\text{column}}=\text{diag}\left(\sum_{i=1}^{n}\Theta_{i:}\right). \end{array}$$

Since the sparse graph obtained by sparse representation is asymmetric, by using the above form, it avoids symmetric processing of the weight matrix of the graph, which is more convenient for understanding, let

(12) $$\begin{array}{c} \text{Lap}=D_{\text{row}}+D_{\text{column}}-\Theta -\Theta^{T},\\ D=D_{\text{row}}+D_{\text{column}}. \end{array}$$

Also adding a constraint, we get

(13) $$\begin{array}{c} P^{T}X\;DX^{T}P=I. \end{array}$$

The formula can be transformed into

(14) $$\begin{array}{c} \underset{p}{\min}\begin{array}{c} Tr\left[P^{T}X\text{Lap}X^{T}P\right]\\ Tr\left[P^{T}XDX^{T}P\right] \end{array}. \end{array}$$

Formula (14) can be solved by generalized eigenvalue decomposition. By generalized eigenvalue decomposition of (*X*Lap*X*^*T*^, *X*  *DX*^*T*^), we obtain the corresponding eigenvalues and eigenvectors. The projection matrix P can be constructed from the eigenvectors corresponding to the smallest *p* eigenvalues, namely,

(15) $$\begin{array}{c} P=\left[v_{1},v_{2},\ldots ,v_{p}\right]. \end{array}$$

*v*_*i*_ is the eigenvector corresponding to the eigenvalue *s*_*i*_, *s*_1_ < *s*_2_ < ⋯<*s*_*p*_. After many iterations, the weight matrix Θ of the sparse graph is stable.

RETRACTED

## 3. Red Wine Flavor Experiment

### 3.1. Experimental Methods and Instruments

The main reagents and instruments of the experiment are shown in Tables 1 and 2:

The paper selects the optimal CAR/PDMS extraction head, and obtains the optimal extraction time and temperature according to the optimal number of peaks and abundance of peaks. The four levels of salt addition (NaCl, W/V) of 10%, 20%, 30%, and 40% were used for univariate analysis to obtain the optimal salt addition.

Gas chromatography conditions: it uses triple quadrupole tandem mass spectrometry (TSQQuantumGC, ThermoFisher Scientific), Q2 selects two chromatographic columns, TR-5MS (30m × 0.25 mm × 0.25 um; (J&WScientific, Folsom, CA, USA), and TR-WAX(30m × 0.25 mm × 0.25 um; (J&WScientific, Folsom,CA,USA). It inserted the SPME fiber tip into the injection hole, desorbed at 250°C for 1 min, and ran the sample for 30 min. The fiber head was kept on the Jack for 5 minutes to remove impurities, the injection hole was in the no-crack mode, 99.9995% helium was passed through for 1 minute, and the flow rate was adjusted to 40 cm/s for the mobile phase of the GC column. The initial temperature of the box is 50°C, 1 min, rise to 100°C at 5°C/min, then rise to 250°C at 10°C/min, and hold for 9 min.

Mass spectrometry conditions: the electron bombardment ionization source (EI+) was selected, the electron multiplier voltage was 350V, the electron energy was 70 eV, and the interface temperature was 250°C. The ion source temperature was 230°C, the scanning mass range was 35–350 m/z, and the scanning rate was 3 Scan/s. It processes data through workstation ThermoXcalibur 2.0 software and workstation.

It uses a hand-held Brix meter for Brix measurement. It first separates the two prisms of the glucometer and wipes the mirrors with deionized water. It then closes the two-sided prism, aligns the glucometer with the light source, observes the reading through the eyepiece, and adjusts the dividing line on the 0 scale. Then it mashes the grapes into juice, and dips two grape juice drops onto the prism with a glass rod. By closing the prism, which points the lens at the light source, it observes the reading through the eyepiece.

### 3.2. Extraction of Red Wine Flavor Substances

In this experiment, the HS-SPME method was used to extract the volatile flavor compounds in grape berries. The grapes used for the optimization experiments were Muscat grapes. The extraction method is to take 100g of frozen mulled grapes and crush them into pulp in a frozen state. It moved the grape berries into a 250 ml beaker, and after sonicating for a period of time, it was refrigerated and centrifuged at 4°C and 7000 r/min for 10 min. A certain amount of the centrifuged supernatant was taken into a 15 mL headspace bottle equipped with a small magnetic stirrer, and a certain amount of NaCl was added to the bottle and sealed. It is adsorbed at a certain temperature for 40 min with different types of extraction heads. After adsorption, the extraction head was inserted into the GC-MS injection port for analysis for 10 min (the injection port temperature was set to 250°C). Because there are many factors that affect the extraction effect, the main aspects of the experiment have been specifically tested and studied. The test methods are as follows.

The fiber coating of different extraction heads is different [16]. Here, four extraction heads of 50/30umCAR/PDMS/DVB, 100umPDMS, 65umPDMS/DVB, and 75umCAR/PDMS are used for comparison, that is, the extraction heads of these four different materials are used, respectively. It adsorbed 8 mL of grape juice added with 3 g NaCl at 40 °C (grape juice was sonicated grape berries for 20 min. The volatile flavor substances in the clarified liquid obtained after being frozen and centrifuged) were kept for 40 minutes each (that is, the extraction conditions were kept the same except for the material of the extraction head). It selects the peak areas of several main volatile flavor substances for comparison, and determines the extraction head with the most suitable adsorption effect.

RETRACTED

Because a large number of volatile flavor substances contained in the peel are difficult to be leached, the method of ultrasonic-assisted leaching was adopted to extract the volatile flavor substances [17]. The ultrasonic time was set as 10 min, 20 min, 30 min and 40 min, respectively. After ultrasonication, the cells were refrigerated and centrifuged at 4°C and 7000 r/min for 10 min, respectively. It was then used a 50/30um CAR/PDMS/DVB extractor to adsorb volatile flavors in 8 mL of clarified grape juice supplemented with 3 g NaCl at 40°C for 40 min. By observing the influence of ultrasonic time on the leaching effect, the peak areas of several main volatile flavor substances were selected for comparison, and the optimal ultrasonic time was determined.

The extraction temperature affects the precipitation of volatile flavor substances, which in turn affects the adsorption effect of the extraction head. Therefore, it is extremely important to choose a suitable extraction temperature. In the experiment, five different temperatures, 30°C, 40°C, 50°C, 60°C, and 70°C, were selected to study the extraction effect [18]. It first ultrasonicated the grape berries for 20 minutes, and then refrigerated and centrifuged them at 4 °C and 7000 r/min for 10 minutes. Then, 50/30 um CAR/PDMS/DVB extraction head was used to adsorb volatile flavor substances in 8 mL of grape juice added with 3 g NaCl at different temperatures for 40 min each. In this paper, the peak areas of several main volatile flavor compounds were also selected for comparison to determine the optimum extraction temperature.

The sample volume affects the distribution balance of the gas-liquid two-phase, thereby affecting the concentration of the adsorbable gas, which in turn affects the detection effect. Therefore, the sample size was also optimized in the experiment. The grape berries were sonicated for 20 min and then frozen and centrifuged at 4 °C and 7000 r/min for 10 min. In this paper, 5 mL, 6 mL, 7 mL, 8 mL, and 9 mL samples were, respectively, taken into 15 mL headspace vials. The 50/30 *μ*m CAR/PDMS/DVB extraction head was used to adsorb the volatile flavor substances in the headspace bottles with different sample amounts of 3 g NaCl at 40°C for 40 min each. In this paper, the peak areas of several main volatile flavor compounds were selected for comparison to determine the optimum sample amount [19, 20].

RETRACTED

The addition of NaCl can increase the ionic strength in the solution and reduce the solubility of some volatile flavor substances in the solution, making it easier to precipitate. Experiments were therefore carried out with different amounts of NaCl to observe its effect on the precipitation of volatile substances. 1 g, 2 g, 3 g, and 4 g of NaCl were used for testing, respectively. First, the grape berries were ultrasonicated for 20 min and then refrigerated and centrifuged at 4°C and 7000 r/min for 10 min. Then, 50/30um CAR/PDMS/DVB extraction head was used to adsorb volatile flavor substances of 8 mL samples with different amounts of salt at 40°C for 40 min. It selects the peak areas of several main volatile flavor substances for comparison to determine the optimum amount of salt added.

### 3.3. Red Wine Flavor

#### 3.3.1. Sensory Evaluation of Red Wine Flavor

Oral saliva is the main physiological component of mouthfeel. Saliva is composed of water (99.5%), proteins (0.3%, mucins, proline-rich proteins, and enzymes) and inorganic substances (0.2%). Mucins are acidic proline-rich proteins, stellate proteins, histidine proteases, and cystine proteases. It binds to the enamel surface, which forms a thin film of saliva. The parotid glands secrete salivary proteins with the ability to bind phenol, and the submandibular and sublingual glands secrete mucins for oral lubrication. In the mouth, ethanol stimulates the tip of the tongue and the trigeminal nerve. Its irritation lasts for a long time, producing a burning, bitter, and sticky feeling. It increases the complexity of the wine body. The presence of ethanol changes the sweetness, bitterness, and strong taste of the wine body, and at the same time interacts with the aroma components and tannins to affect the sensory attributes. Increased ethanol concentration reduces astringency, and ethanol species bind to proteins and polyphenols through hydrogen bonding to enhance viscosity perception [21]. The presence of glycerin can improve the oiliness, body, and persistence of the wine.

Phenolic compounds or polyphenols have aromatic rings carrying one or more hydroxyl groups. Based on the number of phenolic rings and the structure that binds these rings, there are two main classes of polyphenols: flavonoids and nonflavonoids. Taste and texture are significantly affected. Organoleptic properties manifest as astringency, a complex sensation due to epithelial contractions, stretches, or folds. It is generally believed that polyphenolic compounds form complex hydrophobic interactions and hydrogen bonds with salivary proteins (proline-rich proteins). It precipitates salivary proteins and reduces viscosity, and in the rest of the mouth, proline-rich proteins will adsorb to the enamel, creating a “rough” feel. In wine, astringency can be formed by different kinds of compounds (metals, polyphenols, alcohols, and organic acids). It is however mainly related to polyphenols. Different phenolic compounds have different affinities with oral saliva, and the effect of precipitating salivary proteins increases with the increase of the spatial structure complexity of the phenolic ring [22].

RETRACTED

On the basis of single factor optimization of red yeast rice wine with ethanol and reducing sugar content as indicators, sensory flavor evaluation is also used as indicators. It carried out response surface optimization on fermentation time (A), material-water ratio (B), and fermentation temperature (C), and verified the results of single factor analysis of red wine. In this paper, the design expert software is used to analyze the experimental data. It can be seen from Figure 4 that in the response surface test of three factors and three levels, the flavor scores of red yeast rice wine ranged from 70 to 90.

#### 3.3.2. GC-MS Detection

Based on the above optimization experiments on the extraction parameters of HS-SPME, the optimal conditions for the extraction of volatile flavor compounds in grapes were determined. The volatile flavor substances in the mulled grapes were extracted under the optimum extraction conditions. After extraction, the extraction head was inserted into the GC-MS injection port for analysis at 250°C for 10 minutes, and then GC-MS was used for detection. The total ion chromatogram obtained is shown in Figure 5(a). In this paper, the optimal extraction conditions of HS-SPME were also used to extract the volatile flavor compounds in the snake dragon ball grape. It is detected by GC-MS, and the obtained total ion chromatogram is shown in Figure 5(b).

As shown in Table 3, the threshold was set to 17 when analyzing the total ion chromatogram detected by GC-MS. Through database search and analysis, it can be seen that there are 43 kinds of volatile flavor substances, such as alcohols, esters, aldehydes, alkenes, and acids. Among them, hexanal, 2-hexenal, (E)-2-hexenol, and linalool are the most abundant ones, which are the characteristic aroma substances of mulled grapes. During the analysis of the substances, some chromatographic peaks of volatile flavor substances in non-grapes and the siloxane compounds precipitated from the fiber head itself in the extraction head were discarded with confidence below 90%.

RETRACTED

When analyzing the spectrum, the threshold was set to 17, and a total of 22 kinds of volatile flavor substances were detected, including 6 kinds of alcohols, 6 kinds of aldehydes, 5 kinds of esters, 1 kind of phenols, 3 kinds of ketones, and 1 kind of hydrocarbons. The substances with higher content were ethyl acetate at 2.416 min, 2-hexenal at 6.387 min, and 1-hexanol at 7.043 min. At 3.545 min, although the substance content is relatively large, the substance contained in the extraction head. The dibutyl maleate that appeared at 45.950 min is still controversial, not necessarily a volatile flavor substance in grapes, so it is not counted. Volatile flavor compounds in some non-grapes with a confidence level of less than 90% were also discarded. Therefore, the characteristic flavor substances of snake dragon ball grapes are ethyl acetate, 2-hexenal, and 1-hexanol.

#### 3.3.3. Variation Rule of Red Wine Flavor Substances

The changes of succinic acid and acetic acid, tartaric acid, ethyl acetate and ethyl lactate, n-propanol, isobutanol, and isoamyl alcohol are very similar. With the increase of fermentation time, it showed a trend of first increase and then stable. The main organic acid lactic acid is slightly different, showing an upward trend in 1–4d, and a slight decreasing trend in 4–6d. The analysis in this paper shows that Monascus anka has a certain influence on the composition and metabolism of organic acids. It has an enhanced effect on ethyl lactate, but the relative vitality is not high. However, it has little effect on the content and proportion of higher alcohols.

As shown in Figure 6, it can be seen from the fermentation test that in addition to the volatile flavor substances existing in the grape itself. During the winemaking process, the types of volatile flavor substances newly generated by the two grapes are basically the same, but the content is different at different stages. Therefore, it can be proved that the volatile flavor substances newly generated by all grapes during the brewing process (i.e., the fermentation stage, excluding the aging stage) are basically the same, and the brewing experiments of various grapes can also be carried out to accurately prove. When the two kinds of grapes were detected after the fermentation, it was found that the types and contents of the detected substances decreased after 3 minutes, which was too much lower than that in the middle fermentation period. The reason may be that the volatile substances in the fermented wine have indeed decreased or that the flavor substances have evaporated too much during the last detection process, or that the amount of sugar or yeast added at the beginning of the post-fermentation is insufficient, causing the yeast to stop fermenting in the later stage, resulting in the reduction of flavor substances.

RETRACTED

## 4. Resolve and Prediction of Red Wine Multidimensional Spectral Data

### 4.1. Dimensionality Reduction of Multidimensional Spectral Data

The number of projections (*p*), that is, the low-dimensional space dimension, is an important parameter of the dimensionality reduction method, and its value will directly affect the final result. In general, it is hoped that the dimensionality reduction method can make good classification results in very low dimensions. In this experiment, the influence of this parameter on the performance of the algorithm will be directly studied and analyzed. NN classifier is used to handle the classification problem, Dataset(1) randomly selects 10% of the samples as training samples, and Dataset(2) randomly selects 50 samples in each class as training samples. As comparison, all comparison algorithms were also tested under the same conditions. The value of the number of projections (*p*) will vary from 1 to 100 to observe how the performance changes as the parameters change.

The results of the experiment are shown in Figure 7. For all dimensionality reduction methods, when the value of *p* is greater than a certain value, their performance will tend to be stable, and will no longer change greatly with the increase of *p*. Although, the results of the comparison method are stable after the number of projections is greater than 10. However, the sparse graph learning-based method proposed in this chapter achieves a *p*-value of 10 on Dataset(1) and a value of 5 on Dataset(2). Therefore, it can be said that the sensitivity of the algorithm to *p* is equal to or lower than that of the comparison algorithm. Apart from this, another key point is that the results of the proposed method have obvious advantages compared to the comparison algorithms.

### 4.2. Multidimensional Data Spectral Feature Extraction

In order to verify the feasibility of the short-time Fourier transform extraction method in dynamic spectrum extraction, in this paper, a sample is selected and a comparative experiment is performed between the traditional frequency-domain extraction method based on fast Fourier transform (FFT) and the improved frequency-domain extraction method based on short-time Fourier transform (STFT). The analysis band is still 591.85 nm–1119.86 nm. The parameters are set as described above.  Figure 8 is a comparison diagram of the extraction effects of the two methods. It can be seen from the figure that compared with Figure 8(a) and 8(b), it can be clearly seen that the noise is reduced. Dynamic spectral curves improve curve smoothness while maintaining useful information about the original signal.

RETRACTED

### 4.3. PaviaU Experiment

Experimental simulations on PaviaU data have verified the effectiveness of the two methods proposed in this chapter. 40% of the samples are randomly selected as training samples, and the rest are test samples.

It can be seen from Figure 9 that on the PaviaU data, the choice of parameter *k* when constructing the matrix Φ for the overdetermined equation has a certain influence on the experimental results. When *k* = 100, the classification result is the best. And it can be seen that when the number of hidden layer nodes drops to 100, the curve reaches a steady state. Therefore, in the following experiments, in the hidden layer node optimization stage, *k* = 100, and the sparsity is taken as 100.

Figure 9(b) shows the feature selection stage, after taking different k values to construct the matrix Φ. With the different eigenvalues selected, the classification accuracy of the algorithm changes curve. It can be seen that when *k* = 60, the classification result is the best, and it stabilizes when the sparsity is 60. Therefore, in the following experiments, in the feature selection stage, *k* = 60, sparsity = 60.

### 4.4. Hyperspectral Data

In the actual situation, the collected linear hyperspectral signal should have noise, so in order to simulate this real signal, the mixed signal MIX should be noised first, and the noise is 30 dB Gaussian white noise. Get MIXN, MIXN can be imagined as the original signal, we collected in practical applications. In this simulation, the wavelet denoising method is adopted to denoise MIXN, and the denoised signal MIXD is obtained. It can be seen from Figure 10 that a better denoising effect can be obtained by using wavelet denoising. When the noise is 20 dB Gaussian white noise, the following denoising effect can be obtained as shown in Figure 10.

The black is the original MIX signal, and the green is the MIXN signal after adding noise. It can be seen that the red and black curves basically coincide, indicating that the denoising effect is good. Since the effects of 20 dB and 30 dB denoising are very close, and denoising is not the focus of this simulation experiment, therefore, 30 dB Gaussian white noise will be used by default for noise addition in subsequent experiments. Since the four sets of signals are known, the solution pick_res of the abundance value can be reversely solved, that is, the approximate value of the original abundance value pick_na, which can also be regarded as a solution of the equation system, so we can get the results as shown in Table 4.

RETRACTED

It can be seen from the residuals that the difference between the two is very small, that is, when using the correct set of data in the endmember library to solve the abundance value, the solution of the abundance value is very close to the original abundance value. This also provides a possibility for us to judge whether the solution is reasonable: that is, when using a correct set of hyperspectral data to obtain the solution of the abundance value, then use the approximate curve of the original spectrum obtained by them, which should be very close to the original spectrum after denoising.

## 5. Conclusion

The volatile flavor substances contained in grapes and wine are the primary indicators for evaluating the sensory quality of wine, and are also an important factor affecting the quality of wine. The composition and content of volatile flavor substances in different wines are very different, and the different proportions of their content contribute to the different regional flavors of wines. This paper mainly studies the changes of volatile flavor substances in grapes before and after winemaking, and aims to explore the process of grape fermentation into wine. The changes of volatile flavor substances carried by grapes and the changes of volatile flavor substances newly generated in the fermentation process in different periods of fermentation. Finally, the differences of volatile flavor substances in grapes and wine before and after fermentation were compared, and the similarities and differences of various grapes into wine were found. The conclusions of the experiment can provide data support for the future research on specific flavor substances in wine.

## Figures and Tables

**Figure 1:** Aroma transformation of wine.

**Figure 2:** Metabolic pathways of flavor substances during yeast fermentation.

**Figure 3:** Dimensionality reduction process based on sparse learning.

**Figure 4:** Response surface map of the effect of fermentation time, material-water ratio, and temperature on sensory flavor. (a) Fermentation time and material-water ratio. (b) Fermentation time and temperature. (c) Material-water ratio and temperature.

**Figure 5:** Flavor comparison between berries and wine. (a) Total ion current diagram of wine flavor volatiles. (b) Total ion chromatogram of grape berry flavors.

**Figure 6:** Changes in the metabolism of aroma substances. (a) The law of acid metabolism. (b) Changes in lipid metabolism. (c) Changes in alcohol metabolism.

RETRACTED

**Figure 7:** Dimension reduction effect varies with multidimensional spectral data. (a) NN classifier. (b) SVM classifier.

**Figure 8:** Two methods to extract dynamic spectrum renderings. (a) Traditional DS extraction method (FFT-based). (b) Optimizing DS extraction method (STFT-based).

**Figure 9:** The effect of parameter *K* on the performance of the algorithm. (a) Influence of sparsity and parameter *k* on the algorithm performance during hidden layer node optimization. (b) Influence of sparsity and parameter *k* on the algorithm performance during feature selection.

**Figure 10:** Denoising effect graph when the noise is 20 dB white noise.

**Table 1:** Main reagents.

Name of reagent/drug	Manufacturer
Sodium chloride	Tianjin quartz clock factory Bazhou chemical industry branch
High activity dry yeast of wine	Angel Yeast Co., Ltd
Potassium metabisulfite	Shanghai Pinchun biochemical technology co., ltd.
Sodium hydroxide	Tianjin Dongli District Tianda chemical reagent factory
Anhydrous dextrose	Tianjin Damao chemical reagent factory
Copper sulfate	Tianjin Damao chemical reagent factory
Potassium sodium tartrate	Tianjin Damao chemical reagent factory
Refined white sugar	Dalian Keduolin Foods Co., Ltd

**Table 2:** Main instruments.

Instrument name	Manufacturer
GC-MS	Agilent Inc.
Multi-head magnetic heating stirrer	Changzhou Guohua Electrics Co., Ltd
JA203 electronic balance	Shanghai Haikang electronic instrument factory
Electronic balance	Fuzhou Huazhi Scientific Instrument Co., Ltd
Electrothermal blowing dry box	Shanghai-Heng Scientific Instrument Co., Ltd.
Ultrasonic cleaner	Kun Shan Ultrasonic Instruments Co., Ltd
Refrigerated centrifuge	Eppendorf Germany Ltd.
Biochemical incubator	Shanghai Jinghong Test Equipment Co., Ltd.
Fridge	He' nan Xinfei Electrics Co., Ltd
Ph meter	Mettler Toledo Instrument (Shanghai) Co., Ltd.

**Table 3:** Composition of volatile aroma compounds in mulled grapes.

Compound type	Total molecular weight	Average retention time (min)	Relative content (%)	Aroma type
Esters	930	23.6	4	Fruit fragrance, grape fragrance, qu fragrance, and pineapple fragrance
Aldehydes	830	16.4	21	Green grass and apple fragrance, fresh raspberry fragrance, and yellow melon fragrance
Alcohol	1756	27.38	44	Lilac, pepper, light Earth
Acids	170	8.93	0.5	Flavor of acetic acid, fresh orange, and lemon
Alkene	783	18.65	3	Citrus and lemon fragrance
Benzene and phenols	760	23.25	3	Specific fragrance
Ketone	540	40.32	3	Violet and rose fragrance
Other	652	20.32	2	—

**Table 4:** Residuals of abundance values.

	Exhaust nozzle	Skin	Tail flame	Background
Pick_na	0.291	0.3956	0.2759	0.05674
Pick_res	0.2735	0.375	0.2716	0.05636
Residual	0.3199	0.0798	0.6791	0.7822

RETRACTED

## Data Availability

The data that support the findings of this study are available from the corresponding author upon reasonable request.
